This article has been retracted.

# Obesity Mass Monitoring in Medical Big Data Based on High-Order Simulated Annealing Neural Network Algorithm

**DOI:** 10.1155/2021/8336887

**Published:** 2021-11-06

**Authors:** Lijian Ren, Xiaoyu Wu, Kaiqing Zhao

**Affiliations:** ^1^School of Architecture, Tianjin University, Tianjin 300072, China; ^2^Faculty of Art & Science, The University of Toronto, Toronto M1C 1A4, Canada

## Abstract

With the rapid development of information technology, hospital informatization has become the general trend. In this context, disease monitoring based on medical big data has been proposed and has aroused widespread concern. In order to overcome the shortcomings of the BP neural network, such as slow convergence speed and easy to fall into local extremum, simulated annealing algorithm is used to optimize the BP neural network and high-order simulated annealing neural network algorithm is constructed. After screening the potential target indicators using the random forest algorithm, based on medical big data, the experiment uses high-order simulated annealing neural network algorithm to establish the obesity monitoring model to realize obesity monitoring and prevention. The results show that the training times of the SA-BP neural network are 1480 times lower than those of the BP neural network, and the mean square error of the SA-BP neural network is 3.43 times lower than that of the BP neural network. The MAE of the SA-BP neural network is 1.81 times lower than that of the BP neural network, and the average output error of the obesity monitoring model is about 2.35 at each temperature. After training, the average accuracy of the obesity monitoring model was 98.7%. The above results show that the obesity monitoring model based on medical big data can effectively complete the monitoring of obesity and has a certain contribution to the diagnosis, treatment, and early warning of obesity.

## 1. Introduction

In recent years, with the rapid development of information science, the combination of medical treatment and information technology to achieve hospital information construction is of great significance to the improvement of the efficiency of residents' health management and the efficiency of medical treatment [1]. After hospital informatization, there will be a large number of patients and a large amount of disease information, namely, medical big data. In order to make the most of the medical big data, related scholars have put forward the concept of disease monitoring, which is to monitor, prevent, and assist treatment of corresponding diseases based on medical big data. Obesity monitoring is one of them [2]. Obesity monitoring means to collect, check, and analyze data on the long-term dynamic distribution of obesity and internal influencing factors of patients and take measures to prevent and control obesity based on the collected data and analysis results. Obesity monitoring is of great significance for the prevention, treatment, diagnosis, and early warning of obesity. In the past, the BP neural network was generally used for obesity monitoring, but the traditional BP neural network has the disadvantages of slow convergence speed and easy to fall into local optimization, so the monitoring efficiency is low [3]. Simulated annealing (SA) algorithm is a heuristic algorithm, which can describe the annealing process of objects. Simulated annealing algorithm has the function of global optimization, so it is used to optimize the BP neural network and construct the SA-BP neural network algorithm, which solves the defects of the BP neural network, namely, easy to fall into local optimization and slow convergence speed [4]. Finally, based on medical big data and SA-BP neural network algorithm, the obesity monitoring model is constructed to realize the monitoring and prevention of obesity.

Wei et al. [5] used simulated annealing algorithm to design a set of minimum cost routes and solved the capacitated vehicle routing problem with two-dimensional load constraints. Lin et al. [6] proposed a heuristic solution method based on simulated annealing algorithm and then solved the marshalling problem of the railway freight transportation system. Sun et al. [7] used simulated annealing algorithm to optimize the Kriging agent model, so as to realize the crashworthiness optimization of the automobile front end structure. Huang et al. [8] proposed an improved simulated annealing algorithm to deal with the fixed contour plane planning problem of modern buildings. The results show that the algorithm can achieve 100% success rate in any benchmark. In order to improve the control performance of distributed tuned mass dampers (DTMDs), Han et al. [9] used the simulated annealing algorithm optimized by genetic algorithm (GA) to obtain the optimal values of design parameters [10]. The results show that the algorithm can well solve the nonconvexity and multimodality problems of the objective function. Hu et al. [11] studied the screening efficiency of domestic Down's syndrome (DS) based on medical big data, and the results showed that medical big data can improve the screening effect. Li et al. [12] established a pharmaceutical knowledge base model based on medical big data to provide clinicians with reliable and reasonable drug treatment advice. In order to protect the privacy of patients' medical data, Jeon et al. [13] proposed a deep learning framework to prevent the leakage of patients' medical data in various medical platforms. Inomata et al. [14] have developed mobile health applications based on medical big data analysis and proposed solutions for the management and prevention of dry eye disease. Sun et al. [15] used medical big data to study obesity model and build an obesity medical service mode based on medical big data. Research shows that this mode is conducive to the development of medicine. Gao et al. [16] built an optimization model of medical big data flow based on convolutional neural network algorithm (CNN) to predict the network link load. The results show that the prediction accuracy of this method can reach 93%.

It can be seen from the above contents that at present, there are many research studies and applications on simulated annealing algorithm and medical big data, but there are few studies on deep mining of medical information combined with simulated annealing algorithm and medical big data. The innovative contribution of this study is that simulated annealing algorithm is used to optimize BP neural network, SA-BP neural network algorithm is constructed, and the obesity monitoring model is constructed based on SA-BP neural network algorithm and medical big data to realize the monitoring, prevention, and control of obesity.

## 2. Obesity Monitoring Model

### 2.1. Simulated Annealing Algorithm

Simulated annealing algorithm (simulated annealing, SA) is used to imitate the process of a heated solid undergoing cooling until its temperature drops to zero. In this process of change, the local solution is probabilistically jumped out and then the global optimal solution objective function is found [17]. According to the simulated annealing algorithm, the initial temperature is the global maximum temperature. At this time, the solid oscillation is at its largest; that is, the probability of low-energy particles is the smallest; when the object is cooled, the solid gradually finds the best advantage and stabilizes and the probability of obtaining low-energy particles increases. When the temperature of the object drops to 0, the particle with the smallest energy can be obtained from all low-energy particles, that is, to find the optimal solution [18]. The physical process of simulated annealing algorithm includes three stages: heating stage, isothermal stage, and cooling stage. The specific description is as follows: (1) Heating stage: heating the object means, in this process, the particles inside the object can move irregularly and finally in a nonuniform state. Define the initial temperature at this time as *T* and the initial value as *x*. (2) Isothermal stage: the object goes from heating and cooling to isothermal stage means, in this process, a suitable temperature is set, so that the ability of all the particles in the nonuniform state of the object is gradually reduced; when the energy of the particles is at the minimum, it can be judged that the system has reached the equilibrium state. Accept the solution better than the original function by judging the evaluation function or accept the second better solution with the Boltzmann probability function, and gradually reduce the temperature [19]. That is, to reduce the temperature *T*, calculate the new solution *x′*, calculate the evaluation function value, if the relative error Δ*y* <  0, or accept the new solution with Boltzmann probability exp (Δ*y*/T); if accepted, let *x* = *x*′. (3) Cooling stage: in this stage, the object is cooled from isothermal temperature to 0°. In this process, the energy of particles in the system is gradually reduced and the movement of particles tends to be orderly, and particles are finally gradually transformed into a crystal state [20]. Judge whether the temperature drops below *T* min, or if there is no better solution after a large number of consecutive calculations, then the algorithm ends.

The SA algorithm is a heuristic search algorithm [21], which adds a probability function to the hill climbing algorithm, which can converge to the global optimal solution, which makes up for the defect that the hill climbing algorithm is easy to fall into the local optimal solution. There are corresponding variables between the simulated annealing algorithm and BP neural network, as shown in Table 1.

Through Table 1, we can combine and replace the corresponding variables between the simulated annealing algorithm and BP neural network, finally achieve the purpose of combining the two algorithms, complete the optimization of the BP neural network, and realize the construction of SA-BP neural network algorithm.

### 2.2. Demand Analysis of the Obesity Monitoring Model

The obesity monitoring model is divided into the obesity monitoring terminal system, remote service system, data storage system, and business system; The remote service system is used to make suggestions to patients through the data provided by the obesity monitoring terminal system. The data storage system mainly stores the patient's identity, medical history, physical condition, and other information data. The business system is used to serve patients, such as network diagnosis or online registration. The structure of the obesity monitoring model is shown in Figure 1.

According to the model, the main functions of the obesity monitoring model are divided into receiving and sending part, health monitoring part, risk assessment part, information storage part, and so on. The receiving and transmitting part is used to receive the basic information, physiological parameters, and past medical history of the patient. In addition, it also has the function of receiving guidance information from the hospital and transmitting emergency information to the outside world. In the health monitoring part, the physiological parameters such as blood pressure, heart rate, and blood glucose are monitored through sensors and other hardware, so that doctors can judge whether the patient has the risk of obesity or whether obesity has the risk of deterioration. The information storage part stores the medical big data of patients to provide reliable data support for doctors to diagnose and treat patients' obesity.

## 3. Construction of the Obesity Monitoring Model Based on SA Algorithm

### 3.1. BP Neural Network

Artificial neural networks (ANNs) can simulate biological neurons and work by imitating the information transmission mode of biological neurons [22–27]. The structure of biological neurons is shown in Figure 2.

The BP neural network is one of the most common artificial neural networks, which can adjust the weight and threshold of the whole neural network with the help of gradient descent method and backpropagation and finally make the sum of square error of all solutions reach the minimum [28]. The working mode of the BP neural network is accomplished with the help of perceptron, and the working mode of the perceptron is expressed as

(1) $$\begin{array}{c} Z=\left\{\begin{array}{c} 1,\;\text{if }\sum_{j}w_{j}x_{j}\geq b,\\ 0,\;\text{if }\sum_{j}w_{j}x_{j}\leq b. \end{array}\right) \end{array}$$

In formula (1), *Z* is the output value of the perceptron; *x*_*j*_ is the input value; *b* is the threshold value; and *w*_*j*_ is the weight. In training, the training error of the BP neural network can be expressed by a quadratic cost function, such as

(2) $$\begin{array}{c} C\left(w,b\right)\equiv \frac{1}{2n}{\sum_{x}\left\|y_{x}-a\right\|}^{2}. \end{array}$$

In formula (2), *w* is the weight set of neural network; *b* is all offsets; *n* is the number of data input; and *a* represents the output vector when the input value is *x*. The value of *C*(*w*, *a*) will decrease as the gradient decreases. When the value is minimum, the goal of neural network is achieved. Δ*C* shows that for any gradient descent process, there is the following formula:

(3) $$\begin{array}{c} \Delta C\approx \frac{\partial C}{\partial w}\Delta w+\frac{\partial C}{\partial b}\Delta b. \end{array}$$

If the gradient vector is expressed by ∇*C*, there is the following formula:

(4) $$\begin{array}{c} \nabla C\equiv {\left(\frac{\partial C}{\partial w},\frac{\partial C}{\partial b}\right)}^{T}. \end{array}$$

If formulas (3) and (4) are combined, there is

(5) $$\begin{array}{c} \Delta C\approx \nabla C\cdot \Delta v. \end{array}$$

In formula (5), Δ*v* shows the decrease of weight and threshold, and the following formula is satisfied:

(6) $$\begin{array}{c} \Delta v\equiv {\left(\Delta w,\Delta b\right)}^{T}. \end{array}$$

In order to make the descent process of any gradient less than 0 and to ensure that *C*(*w*, *a*) becomes smaller, there is the following formula:

(7) $$\begin{array}{c} \Delta v=-\mu \cdot \nabla C. \end{array}$$

In formula (7), *μ* shows the learning rate set by the BP neural network. The following formula can be obtained by combining the above contents:

(8) $$\begin{array}{c} \Delta C\approx -\mu \cdot {\left\|\nabla C\right\|}^{2}. \end{array}$$

The structure of the BP neural network mainly includes input layer, output layer, and hidden layer, as shown in Figure 3.

In the BP neural network, because it uses the backpropagation and gradient descent method to update the weights and thresholds of the neural network iteratively, the error of network will continue to reduce [29]. But, the BP neural network is a multilayer network structure, each layer of the network has the probability to contain *n* local extrema, and the gradient descent method can easily make the whole BP neural network training error fall into local extremum [30]. In order to avoid the problem of BP neural network falling into local optimal solution in obesity monitoring, simulated annealing algorithm can be used to optimize its calculation.

### 3.2. Construction of the SA-BP Neural Network

The prototype of the simulated annealing algorithm was first proposed by Metropolis, later improved by Kirkpatrick, and successfully applied to the combinatorial optimization algorithm. The main goal of this algorithm is to solve the problem of the optimization process falling into a local minimum and overcoming the dependence of the initial value [31–36]. The simulated annealing algorithm simulates and describes the process of a high-temperature object from a high-temperature state to an isothermal state, from an isothermal state to a cooling state, and finally until it drops to zero. During this change, as the temperature of the object continues to drop, the algorithm randomly searches for the global optimal solution in the combined space of all probabilities [37].

The reason why the simulated annealing algorithm can be applied to optimization problems is mainly due to the relatively high similarity between the physical annealing process and the combinatorial optimization problem. The basic flow of the simulated annealing algorithm is shown in the following, where *k* represents the iterative steps of the algorithm; *d*(*x*) represents the temperature cooling update formula; and *E*(*x*) represents the energy function. It can be seen from the algorithm flow that the algorithm includes two layers of loops. The inner loop represents the random search of the state at the same temperature, while the outer loop is the change when the temperature drops and the algorithm stops conditions [38]. According to this characteristic, SA can help the neural network jump out of local optimum. When the temperature is t0, the state of the particles is shown in

(9) $$\begin{array}{c} P\left[E=E\left(r\right)\right]=\frac{1}{Z\left(T\right)}\exp\left(-\frac{E\left(r\right)}{K_{b}T}\right). \end{array}$$

In formula (9), *E*is a random variable of the energy of a molecule, *E*(*r*) represents the energy of the state *r*, *Z*(*T*) represents the normalized factor of the probability distribution, *T* indicates the temperature, and *K*_*b*_ represents the Boltzmann constant. *Z*(*T*) satisfies

(10) $$\begin{array}{c} Z\left(T\right)=\sum_{S\in D}\exp\left(-\frac{E\left(s\right)}{K_{b}T}\right). \end{array}$$

By combining formulas (9) and (10), the probability difference of two particles with different temperatures can be obtained. If *D* represents a state space, it is the set of states with the lowest energy, and *t* is the temperature. In simulated annealing algorithm, the process of a particle randomly selecting a particle around it is a random disturbance and the process of random disturbance is expressed as

(11) $$\begin{array}{c} f\left(x+1\right)=g\left[f\left(x\right)\right]. \end{array}$$

In formula (11), *f*(*x*) represents the current particle; *f*(*x*+1) represents the particle after random disturbance; and *g*(*x*) represents the way to represent random disturbances. In the process of random disturbance, the state of particles before and after disturbance obeys Markov state distribution, so when the temperature is the same, the number of particle search processes can be set as Markov chain length L [39]. It can be seen from Table 1 that the BP neural network and simulated annealing algorithm have commonness and similar characteristics, so they can be combined to build the SA-BP neural network. The weight and threshold of the neural network are adjusted by combining the gradient descent method and random disturbance. The variable replacement method of the SA-BP neural network and simulated annealing algorithm in this method is shown in Table 2.

Then, the training process of SA-BP neural network is as follows: construct the BP neural network and set various parameters; set the initial temperature *T*_0_ of SA algorithm and the way to reduce the temperature; the BP neural network is trained at *T*_0_ time; and the gradient descent method is used to obtain the local optimal error. The BP neural network is randomly perturbed and trained by the gradient descent method to judge the training accuracy of the neural network. The new temperature is obtained by cooling down, and the training is repeated until the accuracy reaches the target error. The training process is shown in Figure 4.

According to the above content, we can complete the construction of SA-BP neural network and then build a obesity monitoring model to monitor obesity.

### 3.3. Similarity Calculation of Obesity

Obesity's damage to the body is mainly manifested in that obesity increases the risk of cardiovascular disease, cerebrovascular disease, and diabetes. According to authoritative statistics released by the Department of Disease Control of the Ministry of Health, the number of overweight and obese people are higher than the number of normal-weight people. The risks of blood pressure, hypertriglyceridemia, high-density lipoprotein cholesterol reduction, and atherosclerosis are several times higher. Some studies have analyzed 32,000 individuals through genome-wide association analysis, screened out a large number of obesity-related mutations, and obtained 6 new obesity genes. The six genes are TMEM18, KCTD15, GNPDA2, SH2B1, MTCH2, and NEGR1.

Therefore, it is possible to use the medical big data of genetic composition such as TMEM18, KCTD15, GNPDA2, SH2B1, MTCH2, and NEGR1 in the patient's body to predict and monitor obesity.

Through the follow-up forest algorithm, the key obesity index (BMI index) is used as the dependent variable and the carrying status indicators of TMEM18, KCTD15, GNPDA2, SH2B1, MTCH2, and NEGR1 are used as independent variables to perform factor importance analysis. Taking the physiological data of this case study case as the data set, after calculation, carrying status of the TMEM18 gene is the most important for obesity, followed by the GNPDA2 gene. In order to simplify the subsequent modeling and calculation process of the SA-BP neural network, the TMEM18 index is identified as a strong correlation index for patient obesity and the functions of the TMEM18 gene are similar between the same or similar diseases. Therefore, sorting out and analyzing the information transmitted by the TMEM18 gene can help in monitoring obesity. Based on the similarity calculation method, construct similarity data to study the relationship between obesity and TMEM18 gene, use these sample data to train the SA-BP neural network, and perform deep learning, so as to achieve the purpose of predicting and monitoring obesity [36]. At present, the main calculation methods of the correlation between obesity are the semantic similarity of obesity based on semantic correlation and the functional similarity based on gene correlation. Among them, the semantic similarity can be calculated by constructing a directed acid graph (DAG) based on the basic classification information of the disease. For obesity *D*, the DAG diagram is obtained according to medical big data and its semantic value is defined as

(12) $$\begin{array}{c} DV\;1\left(D\right)=\sum_{d\in T\left(D\right)}1\left(d\right). \end{array}$$

In formula (8), T(D) is the set of all nodes in the DAG graph of disease D. Then, the contribution of disease *d* to the semantic value of *D* is expressed as follows:

(13) $$\begin{array}{c} D_{D}1\left(d=1\right),\;\text{if }d=D,\\ D_{D}1\left(d\right)=\max\left\{\Delta *D_{D}1\left(d^{\prime }\right)|d^{\prime }\in \text{children of }d\right\}\text{,}\;\text{if }d\neq D. \end{array}$$

In formula (13), *d* is calculated as follows: Then, the semantic similarity between the two diseases *d*(*i*) and *d*(*j*) is calculated as follows:

(14) $$\begin{array}{c} SS\left(d\left(i\right),d\left(j\right)\right)=\frac{\sum_{t\in T\left(d\left(i\right)\right)\cap T\left(d\left(j\right)\right)}\left(D_{d\left(i\right)}1\left(t\right)+D_{d\left(j\right)}1\left(t\right)\right)}{DV\;1\left(d\left(i\right)\right)+DV\;1\left(d\left(j\right)\right)}. \end{array}$$

According to the above content, the semantic similarity between obesity genes can be calculated. When the functional differences between the two TMEM18 genes are large, there will be few diseases associated with them. On the contrary, there will be more diseases associated with them. Therefore, we can predict and monitor obesity according to the functional similarities between TMEM18 genes. TMEM18 genes and disease networks are shown in Figure 5.

According to Figure 5, TMEM18 genes with functional similarity are associated with semantically similar diseases. According to the similarity between TMEM18 gene and disease, we can calculate the similarity between each pair of TMEM18 gene and the TMEM18 gene and then get a TMEM18 gene functional similarity matrix FS, which is called TMEM18 gene functional similarity method (MISIM).The calculation method of FS is shown in

(15) $$\begin{array}{c} FS\left(i,j\right)=\frac{\sum_{1<i<m}S\left(d_{i},D_{2}\right)+\sum_{1<i<n}S\left(d_{i},D_{2}\right)}{m+n}. \end{array}$$

Formula (15) represents the number of diseases, and the relevant data of the functional similarity matrix can be obtained through medical big data. According to the above content, we can obtain obesity data samples with similar characteristics, then train the obesity monitoring model, and finally realize the monitoring of obesity.

## 4. Performance Analysis of the Obesity Monitoring Model

### 4.1. SA Algorithm for BP Neural Network Optimization Effect Analysis

In order to verify the optimization effect of simulated annealing algorithm on the BP neural network, the SA-BP neural network and BP neural network are constructed. After extracting the feature subset from the same medical big data samples, the SA-BP neural network and BP neural network are trained. The redundancy rate of the feature subset is shown in Figure 6.

It can be seen from Figure 6 that the redundancy rate of the feature subset decreases with the increase in the number of features, indicating that it can be used. The training times of the SA-BP neural network and BP neural network to achieve the target accuracy are compared by using the above feature subset. The training times required for the SA-BP neural network and BP neural network to achieve the same target accuracy are shown in Figure 7.

As can be seen from Figure 7, the SA-BP neural network needs 500 training times to reach the target accuracy (0.0001), while the BP neural network needs 1980 times to reach the target accuracy, 1480 times more than those of the SA-BP neural network. The above results show that the training times of the SA-BP neural network to achieve the same target accuracy are much less than those of the BP neural network, indicating that the training efficiency of the SA-BP neural network is higher, indicating that simulated annealing algorithm can optimize the BP neural network well. Using the above data, the prediction accuracy of the BP neural network and SA-BP neural network is tested, as shown in Figure 8.

As can be seen from Figure 8, the prediction accuracy of the SA-BP neural network is constantly improving with the increase in the number of features, up to 79.7%, while the accuracy of the BP neural network is up to 53.4%, 26.3% lower than that of SA-BP neural network. The SA-BP neural network and BP neural network are used to predict and monitor the same data samples, and the results are verified with the real results in the past. The mean square error (MSE) and mean absolute error (MAE) are used to express the error between the predicted value and the real value of the SA-BP neural network and BP neural network. The mean square error and mean absolute error of the SA-BP neural network and BP neural network are shown in Table 3.

It can be seen from Table 3 that the mean square error of the SA-BP neural network for sample data prediction is 1.77, the mean square error of the BP neural network for sample data prediction is 5.20, and the mean square error of the BP neural network is 3.43 higher than that of the SA-BP neural network. The average absolute error of the SA-BP neural network is 0.09, the average absolute error of the BP neural network is 1.90, and the average absolute error of the BP neural network is 1.81 higher than that of the SA-BP neural network. From the above content, it can be seen that the mean square error and absolute mean error of the SA-BP neural network are significantly lower than that of the BP neural network, indicating that the accuracy of the SA-BP neural network is higher than that of the BP neural network and the optimization effect of simulated annealing algorithm on BP neural network is better.

### 4.2. Monitoring Error Analysis of the Obesity Monitoring Model

The monitoring accuracy of the obesity monitoring model is an important standard to evaluate the practicability of the obesity monitoring model. In order to obtain the monitoring error of the obesity monitoring model, the SA-BP neural network is used to construct the obesity monitoring model. The obesity monitoring model is trained by the data samples with obesity characteristics. Then, the obesity monitoring model is used to monitor *n* groups of sample data. Finally, the output value of the model is compared with the real value. The output error of the obesity monitoring model is shown in Figure 9.

As can be seen from Figure 9, with the change in temperature, the output error of the obesity monitoring model also changes. When the temperature is 75°C, the output error of the obesity monitoring model reaches the highest, which is 3.2. When the temperature is 65°C, the output error of the obesity monitoring model is the lowest, which is 1.79. When the temperature is 0°C, the output error of the obesity monitoring model is 1.87. When the temperature is 100°C, the output error of the obesity monitoring model is 2.84. Overall, the average output error of the obesity monitoring model is 2.35. The above results show that the output error of the obesity monitoring model is small, which is close to the actual value and has high practicability.

### 4.3. Accuracy Analysis of the Obesity Monitoring Model

The SA-BP neural network was used to establish the obesity monitoring model. Based on medical big data mining, the complexity of the model is calculated. The data with obesity characteristics were used as training data samples to train the obesity monitoring model. The obesity monitoring model after training was used to monitor four groups of sample data. The differences between the monitoring results and the actual results were recorded and compared to evaluate the monitoring accuracy of the obesity monitoring model. The difference between the monitoring results of the obesity monitoring model and the actual results of the four groups of sample data is shown in Figure 10.

It can be seen from Figure 10 that the average monitoring accuracy of the obesity monitoring model is 98.7%, which indicates that the monitoring accuracy of the obesity monitoring model can meet the actual needs and has high practicability.

## 5. Conclusion

With the development of information technology, disease monitoring has become a research hotspot. In this paper, we use simulated annealing algorithm to optimize the BP neural network and build high-order simulated annealing neural network algorithm. Based on medical big data, we use high-order simulated annealing neural network algorithm to build the obesity monitoring model, so as to realize the monitoring and prevention of obesity. The results show that the SA-BP neural network needs 500 training times to reach the target accuracy (0.0001), while the BP neural network needs 1980 training times to reach the target accuracy, 1480 times more than those of SA-BP neural network. The mean square error of the SA-BP neural network is 1.77, the mean square error of the BP neural network is 5.20, and the mean square error of the BP neural network is 3.43 times higher than that of the SA-BP neural network. The average absolute error of the SA-BP neural network is 0.09, the average absolute error of the BP neural network is 1.90, and the average absolute error of BP neural network is 1.81 times higher than that of the SA-BP neural network. With the change in temperature, the output error of the obesity monitoring model also changes and the average output error is 2.35. After training, the average accuracy of the obesity monitoring model was 98.7%. The above results show that, compared with the traditional obesity detection methods, the obesity monitoring model in this paper has higher monitoring and prediction accuracy, lower error, and higher practicability. At present, there is no in-depth research on disease similarity calculation, which needs to be further improved.

## Figures and Tables

**Figure 1:** Structure diagram of the obesity monitoring system.

**Figure 2:** Structure of the biological neuron.

**Figure 3:** Structure diagram of the BP neural network.

**Figure 4:** Training process of the SA-BP neural network.

**Figure 5:** TMEM18 genes and disease networks.

**Figure 6:** Feature subset redundancy rate.

**Figure 7:** Performance comparison between the SA-BP neural network and BP neural network.

**Figure 8:** Prediction accuracy of the BP neural network and SA-BP neural network.

**Figure 9:** Output error of the obesity monitoring model.

**Figure 10:** Monitoring accuracy of the obesity monitoring model.

**Table 1:** Variables corresponding to the simulated annealing algorithm and BP neural network.

-	Algorithm	
	BP neural network	Simulated annealing
Corresponding variable	BP neural network with specific weights and thresholds	Particle state at a specific temperature
	Prediction error under specific weight and threshold	Particle state energy at a specific temperature

**Table 2:** Variable replacement of the BP neural network and simulated annealing algorithm.

SA	Replace with	SA-BP neural network
Markov chain length		1
Particle state energy at a specific temperature		Training error
Temperature reduction times		Random disturbance times

**Table 3:** Prediction error of the SA-BP neural network and BP neural network on sample data.

Neural network	BP neural network	SA-BP neural network
MSE	5.20	1.77
MAE	1.90	0.09

## Data Availability

The data used to support the findings of this study are available from the corresponding author upon request.
